This article has been retracted.

# Biochar-based compost: a bibliometric and visualization analysis

**DOI:** 10.1080/21655979.2023.2177369

**Published:** 2023-04-27

**Authors:** Sinazo Ajibade, Ebenezer C. Nnadozie, Chuleemas Boonthai Iwai, Suresh Ghotekar, Soon Woong Chang, Balasubramani Ravindran, Mukesh Kumar Awasthi

**Affiliations:** a Department of Agronomy, Faculty of Science and Agriculture, University of Fort Hare, Alice, South Africa; b Department of Soil Science, Institute of Environmental Sciences, Hungarian University of Agriculture and Life 13 Sciences, Gödöllő, Hungary; c Whyte & Rhyte Creative Solutions Ltd, Lagos, Nigeria; d Integrated Land and Water Resource Management Research and Development Center in Northeast Thailand, Khon Kaen University, Thailand; e Department of Chemistry, Smt. Devkiba Mohansinhji Chauhan College of Commerce and Science, University of Mumbai, Silvassa, India; f Department of Environmental Energy & Engineering, Kyonggi University, Suwon-si, Gyeonggi-do, Korea; g College of Natural Resources and Environment, Northwest A&F University, Yangling, Shaanxi, PR China

**Keywords:** Biochar, compost, biochar-compost, soil, plant, bibliometric analysis

## Abstract

The co-application of biochar compost as organic amendment for crop production and soil remediation has gained momentum due to their positive effect on plant growth and soil quality improvement. The application of biochar and compost which are green and cost-effective soil remediators would promote the availability and distribution of food, planetary conservation, alleviate poverty, and enhance the attainment of Sustainable Millennium Development Goals (SDGs). A bibliometric analysis was conducted to overview research on biochar compost from 2011 to 2021. Two hundred and fifty-four research papers were retrieved from the Scopus database and analyzed using VOS viewer. Analysis revealed that 217 (85.43%) were articles, 21 (8.27%) were conference papers, and 12 (4.72%) were review papers. The results showed an exponential increase in the number of publications. The most productive countries in the investigated subject were China (49), followed by USA (36), Australia (29), Italy (28), Germany (25), and Indonesia (20). After the search terms, ‘soil,’ which had links with keywords like ‘soil fertility,’ ‘soil quality,’ ‘soil pollution,’ ‘phosphorus,’ ‘nitrogen,’ ‘maize,’ ‘greenhouse gas,’ etc., had the highest occurrences (94). From the results of the current hotspot research in the field, the effect of biochar-compost mixture and co-composted biochar on soil remediation is currently being studied by several researchers. Biochar and compost incorporation in soil reduce the uptake of pollutants by plants which consequently increase essential nutrients for plant and soil productivity.

## Highlights

● Biochar-compost research has been increasing for the past eleven years

● China is most productive country in biochar and compost application

●Biochar-compost and co-composted biochar are effective elixirs for soil amendment and nutritional enrichment

## 1. Introduction

As the United Nations (UN) predicted, the world population, with a staggering 7.7 billion in 2019, will be 8.5 billion by 2030 [1] [2]. Africa is projected to account for over 50% increase in world population between 2020–2050; in contrast, China, the most populous nation globally, is expected to have population losses within the same period [3]. Africa and Asia are the continents with the highest number of poverty-infested populations [4; 5]. Around the world, 4973.4 million hectares of land are available for agricultural purposes [6]. Europe, America, and Oceania occupy the least of this portion at 9–12%; the most extensive agricultural lands are available in Asia (38%), while Africa occupies the midpoint at 23% [7]. However, arable lands are declining due to land degradation, residential purposes, drought, advancement in science and technology, and natural and human-induced disasters [8; 9].

These would adversely affect the availability of agricultural land, food distribution, and climate change, which threatens the ecosystem. Together with United Nations Sustainable Development Goals (UNSDGs) and the conservation of the planet, land reclamation, protection, and nourishment are critically necessary to accommodate a rising population. Based on [10] safe recycling of organic biological waste for sustainable management and reclamation of degraded soil may help achieve the UNSDGs. Contrary to the effect of chemical fertilizers on soil degradation with a negative effect on sustainable agriculture [11; 12], organic fertilizers have a prolonged positive impact on soil fertility and are safe [13; 14]. There has been increasing interest and research in applying compost, biochar, and the mixture of biochar compost to nourish agricultural soil. Biochar is the deposit from biomass carbonization at high temperatures in a controlled air environment [15]. The biochar’s unique properties, like surface functional groups, specific surface, and pore openings, depend on the biomass’s nature and nurture. Similarly, compost is a mixture of organic materials that have undergone a natural decomposition process [16].

The low cost of biochar promotes its multifunctional application in science and technology. When incorporated into animal feed, biochar aids digestion; feces from animals fed with biochar constituted meals have less odor and can be used as organic manure [17]. Biochar is a good candidate for the design of slow-release fertilizers [18]; such fertilizers will reduce cost, loss of profitable work time, and wastage. In the food industries, biochar has been adapted to design biodegradable packaging materials for perishable agricultural products [19]. Such packaging materials increase the shelf life of perishable food products; biodegradable package materials promote green science and technology. In the built environment and engineering sector, the utilization of biochar in the preparation of mortar reduces the amount of sand and cement required for the mixture [20]. The sequestration of heavy metals and dyes from industrial and hazardous wastes via adsorption on biochar is a low-cost and relatively cheap green remediation technique [21–23]. The adsorbed metals can be treated and re-used accordingly.

The combined co-application of biochar and compost to agricultural soils has been increasing in research trends, including the application of co-composted biochar as a final product from the addition of biochar to raw composting materials for plant growth and improved soil quality [24; 25], and for the treatment of soils polluted with inorganic and organic contaminants [26; 27]. The increased attention is due to the favorable physicochemical properties [28], and biological properties [29; 30]. It should be noted that three approaches are used for the co-application and the production of biochar-compost, and these include (i) mixing of biochar with compost after composting process followed by its application to soil, (ii) addition of a known amount of biochar to raw materials at the beginning of the decomposition process before soil application [31], (iii) incubation of compost and biochar to a specific time before soil application. The biochar compost produced in (ii) and (iii) is referred to as incubated compost or co-composted biochar, respectively.

The current bibliometric analysis critically examined the biochar-based compost for agricultural purposes. Bibliometric analysis is an important tool for quantitative analysis that has been used in various fields to effectively analyze field development or the overall trend of a subject [32]. To understand the current research trends on the topic, VOS viewer, an information visualization software, was used to analyze the data retrieved from the Scopus database between 2011 to 2021.

## 2. Literature search

### 2.1. Biochar compost mixture

For many years, compost has been used as a natural soil amendment to enhance crop yield [33]. Based on [34] the components of biochar and compost show a synergistic effect, as they enhance each other’s properties, with their combined influence on crop growth and quality. In recent studies, biochar has been combined with finished compost [35–37] to achieve a synergistic effect. Table 1 represents recent studies and their results on the effect of biochar mixed with final compost, and co-composted with raw compost material on soil fertility and plant growth. For instance [36], conducted a two-year field study, on the effect of the combined application of biochar and finished compost at an application rate of 5 t ha^−1^ on soil nutrient profile and maize (*Zea mays*) yield. The feedstock used was cow manure for both biochar and compost. The authors reported an 80.52% increase in soil organic matter, a 0.96%, 12.53 mg kg^−1^, and 208.33 mg kg^−1^ increase in total N, soil available P, and extractable K content respectively; in the treatment with both biochar and compost. The pH of the calcareous soil used in their study declined from 7.8 to 6.8, and the decline was associated with the increasing availability of P in the soil after combined application with biochar and compost due to changes in soil pH and amelioration of Ca^2+^. Compared to the control treatment, agronomic effects of biochar and compost on maize yield were reported on the increased 1000 grain weight (14.70%), plant height (43.23%), harvest index (9.90%), including an increase in biological and grain yield (13.44% and 46.29%). While a significant increase in grain N (51.2%), P (48.14%), and K (3%), and the highest shoot P-value of 3.20 g kg^−1^, and a K content of 16.80% compared to the control treatment were reported.

**Table 1.** Recent papers on the interactive effect of biochar and compost on soil fertility and crop yield.

*Biochar*	*Compost*	Application rate	Test crop	Soil type	Effect on soil fertility	Effect on crop growth	References
**Biochar-Compost source**							
Cow manure		5 t ha^−1^	Maize (*Zea mays*)	Calcareous soils	Increased soil organic carbon, N, soil available P, and extractable K, reduced soil pH	Increased grain yield, plant height, biological yield, 1000 grain weight, harvest index, shoot and grain N, P, and K	[36]
Argan shells waste	Varied vegetable organic matter	2% 4% 6%	Quinoa (*Chenopodium quinoa*), Alfalfa (*Medicago sativa*) and Sugar beet (*Beta vulgaris*)	Alkaline soil	Increased N, P, CEC, total organic matter, K, Na, Ca, and Mg	A significant increase in plant biomass for quinoa at the biochar-compost application rate of 6%, and a significant increase at an application rate of 4% for Alfalfa.	[38]
Oil palm kernel	Food waste	-	*Cordyline fruticosa*, *Coleus* sp., and *Rhoeo discolor*	3: 2: 1 (topsoil: black organic soil: sand	The results showed no significant differences in soil pH, organic matter, and total nitrogen for each plant species after the application of biochar and compost	After the treatment with biochar and compost and <20% fertilizers, the results showed increased total biomass of *Coleus sp*, with the same trend observed in plant height results of Cordyline sp.	[39]
Cacao shell	manure	20 t ha^−1^	Cayenne pepper (*Capsicum frutescens L*.)	Acid upland soil	Biochar and compost did not dhow significant effects on soil physicochemical properties	The combined biochar and compost had positive effects on plant canopies, fresh fruits, and plant height 10 weeks after planting	[40]
Hardwood	Chicken manure	4%	Chinese cabbage (*Brassica Rapa, Chinensis Group*), Papaya (*Carica papaya cv Sunrise*)	Andisol Oxisol	Soil pH of both soils increased, including total N, extractable P, Mg, and Ca when biochar and compost were incorporated, and surface supplied at 0–10 cm soil layer.	The biomass of both Chinese cabbage, and Papaya increased by more than 10% when biochar and compost mixture was incorporated, and surface applied.	[41]
**Co-composted Biochar**							
Rice husk	Poultry litter	10 Mg ha^−1^	Maize (*Zea mays*)	Oxisol	Increased soil organic matter	Higher plant height Higher aerial portion Higher chlorophyll content	[42]
Poultry litter	geranium waste, soil, and mature compost	0 t ha^−1^ 5 t ha^−1^ 10 t ha^−1^	Eggplant (*Solanum melongena L.)*	Torripsamments, siliceous, hyperthermic	Increased soil organic matter, N, P, field capacity, useful pores, water-holding pores, available water, and soil biota (bacterial cells)	Enhanced eggplant growth and productivity Increased chlorophyll content, stomatal conductance, and photosynthetic efficiency	[43]
Industrial hemp (*Cannabis Sativa)*		10% 20% 40% 80% 100%	*Ocimum basilicum*	Commercial garden soil	-	Increased seed germination, fresh weight, and percentile of plant height at 10% and 20% co-compost biochar application rate, with no significant differences to crops planted in soil alone	[44]
Cotton (*Gossypium hirsutum* L.) stalks		2.5 t ha^−1^	Maize (*Zea mays*) and Cotton (*Gossypium* spp.)	Lixisol	Improved soil properties	Higher grain yield of maize and cotton	[45]
Produced by Zhejiang Raymond Agricultural Polytron Technologies Inc. (Hangzhou, Zhejiang), with no information about feedstock		0% 1% 3% 5%	*Tetrastigma hemsleyanum* Diels & Gilg	Medium-thick yellow-brown earth	Significant increase of soil pH, total N, and P, and soil organic matter, in the treatment with 5% co-composted biochar	Increased total *T. hemsleyanum* biomass in the following order: 3% > 1% > 5%	[30]

[41] using Andisol and Oxisol with a pH of 6.0 and 6.9, conducted a pot trial to investigate the effect of incorporated and surface applied mixture of biochar produced from hardwood and compost from chicken manure at an application rate of 4% (v/v) on soil fertility, papaya (*Carica papaya cv Sunrise*), and Chinese cabbage biomass (*Brassica Rapa, Chinensis Group*). The incorporation and surface application of the mixture resulted in higher extractable P, N, Ca, and Mg. The authors also reported increased plant biomass in both tested crops. Between the two soil types, a greater response in terms of improved soil pH, root biomass, and plant nutrient uptake was reported in acidic Andisol than the Oxisol. The results of these studies [36; 41], show that the mixture of biochar and compost in soils with deficient P like Andisol [46] and calcareous [47] soils can be improved. For instance [48], reported that biochar and compost might be the source of available and exchangeable P either by making native P available or through direct application. Also, in an earlier study by [49] co-application of biochar and compost produced from agro-industrial wastes was used to enhance the P availability in acid soil. The authors reported increased available P, total P, organic P, and inorganic P fractions, and associated their findings with increased pH, and reduced exchangeable iron, aluminum, and acidity in the soil. Also, nitrogen (N) content was increased, and based on [50], the mixture of biochar and compost as a soil amendment, improves N use efficiency and prevents N immobilization. As an essential element, N promotes plant metabolisms, and growth, including the creation of chlorophyll content for agricultural yields.

### 2.2. Co-composted biochar

In numerous studies, the effect of co-composted biochar on the fertility of soil and crop productivity has shown a great potential of the material to enhance soil fertility and crop productivity. For example, in the study of [42] the effect of co-composted biochar on the properties of an Oxisol (pH = 4.51) and maize growth was investigated at different application rates. The authors observed increased soil pH of between 0.70 and 0.73, increased aerial portion (7.8% to 108.2%), plant height (46.86% to 25.74%), with increased chlorophyll content, plant nutrient content, and soil organic matter which increased with the biochar ratio of the co-composted biochar. Based on the observation of [51] the application of co-composted biochar enhances the water retention capacity of sandy soils compared to compost without biochar. Even under salt-affected soils, the application of co-composted biochar increases soil properties, plant growth, and water use efficiency. For example [43], stated that the amendment of soil with cocomposted poultry litter biochar at three application rates (0, 5–10 t ha^−1^), and under different irrigation regimes (60, 80, and 100 of crop evaporation rate (ETc)) resulted in increasing the productivity, leaf area, leaf number per plant, dry weight, the stem of the diameter of eggplant, including increased chlorophyll content, stomatal conductance, and photosynthetic efficiency of water-stressed eggplant at 80% ETc. The authors associated their findings with increased soil properties such as hydraulic conductivity, pH, EC, bulk density, water-holding pores%, useful pores%, fine capillary pores%, available water, and soil biota after the application of co-composted biochar to salt-affected soils. Interestingly, the utilization of biochar can improve animal waste composting when done at an application rate of 5–10% [29,52]. In the study of [29] the application rate of 10% enhanced the organic matter degradation and reduced greenhouse gas emissions and ammonia, while [52]observed reduced emissions of NH_3_ by 30% and 44%. The highest application rate could induce desiccation in composting due to excess aeration [53]. It is worth noting that, the cost of producing co-composted biochar is lower than the incubation mixture of biochar and compost [54] since the combination of biochar and compost involves composting, and subsequent incubation which are two separate processes.

### 2.3. Application of biochar, compost, and co-composted biochar on soil remediation

Even though compost has high nutrient content (e.g. N, K, P, Mg or Na, and Ca), increasing microbial activity and soil enzymes [55], however, the nutrients that are rapidly released into the soil reduces its efficiency as a fertilizer [56], and is a threat to environmental pollution. The effect on environmental pollution associated with the inorganic and organic contaminants contained in the compost [57] might pollute the soil after its application. Owing to large cation exchange capacity and abundant functional groups [58; 59], biochar has considerable adsorption capacity for organic contaminants (like PAHs) and heavy metals and can, therefore, immobilize organic contaminants and heavy metals from the compost. Based on the observation of [56] biochar contains residues of PAHs, as a byproduct of the pyrolysis process, and these include among others perfluorooctanesul- phonic acid (PFOS), perfluorooctanoic acid (PFOA), furans (PCDD/F), and dioxins. However, PAHs in biochar were decreased in biochar-based composting, which according to [60]was associated with a large amount of fungi responsible for the degradation of PAHs. Hence, research on the co-application of biochar and compost for soil remediation has gained momentum.

The hyphenated application of biochar and compost for heavy metals contaminated wetland has been reported by [61]. Different constituted ratios of biochar and compost were investigated for the remediation of heavy metals, and it was discovered that higher pH was obtained when biochar addition was 20 and 40%. In their study, all amendments studied significantly showed reductions in soil Cd and Zn. The mechanisms by which biochar and compost stabilize heavy metals in contaminated soils are shown in Figure 1. The removal of contaminants is moderated by the interaction of functional groups on both the analytes and the biochar. These functional groups such as OH, COOH, and NH interact primarily through the physisorption process to form a hydrogen bond, π-π interaction, and complexation. The products from the chemical interactions are less toxic than their default forms. Based on the findings of [62] the biochar-constituted soil was effective for the uptake of Cd, Ni, Cu, Zn, and Pb via ion exchange, electrostatic attraction, and surface complexation. Similarly, nonpolar organic compounds were remediated through hydrophobic effect, partition, and pore filling, while polar organics were cleared by electrostatic attraction, hydrogen bonding, surface precipitation, and specific interaction.

**Figure 1.** Mechanisms in which biochar and compost stabilize heavy metals in contaminated soils. **Source**: Own representation.

The mechanisms explain that the divalent cations such as Pb (II), and Cd (II) are readily exchanged with elemental Ca^2+^ in the soil and compost. The uptake of toxic Cr (VI) is preceded by attraction to Fe^3+^ in the compost, followed by reduction by zero-valent iron Fe (O) to less toxic Cr (III) which is cleared via ligand exchange by N-H and C-O functional groups. Benzene and phenyl compounds are adsorbed via pi-pi bond interaction. Cu^2+^ would readily form chelate or complex with the OH groups on the biochar and compost (Figure 1).

## 3. Materials and methods

The data on the biochar-based compost was retrieved from Scopus, a citation and abstract academic database launched in 2004 by Elsevier. Scopus is an exhaustive summary and citation database with millions of records from journals, conference proceedings, and books. Based on [63] the database has more than 22 600 peer-reviewed titles, more than any other academic database. The search terms used were ‘biochar and compost’ OR ‘biochar compost.’ Of the 254 publications, 231 were from journals, 18 from conference proceedings, and 5 from book series. Of the retrieved document, 245 were in English, 8 in Chinese and 1 in Hungarian.

### 3.1. Analysis tools

A bibliometric analysis was used for the literature review. In the present study, 254 publications were selected after data refinement, and based on [64] the bibliometric analysis is recommended if at least 200 publications are available for review. One of the advantages of using bibliometric analysis includes the following; (i) bibliometric analysis is widely used in developing the whole subject field [65] and hotspot research [66], (ii) the analysis uses quantitative analysis and statistical analysis to research knowledge structure and research field development, (ii) the construction of a network based on the relationship between countries or co-authorship, authors, organizations, journals [67], including keywords about the field, is possible with the bibliometric analysis [68]. The stages of bibliometric analysis used in the present paper are shown in Figure 2. Stages included in step 5, such as performance analysis, bibliometric mapping, and network, were used. Based on [69] performance analysis focuses on the productivity and impact of biochar and compost publications, while the scientific mapping searches for research themes within biochar and compost literature. The total number of publications, citations, and h-index under performance mapping was evaluated as part of the descriptive analysis. The h-index is measured using Equation 1.

1 $$h-index\left(f\right)=\max\left\{i\in N:f\left(i\right)\geq i\right\}$$

**Figure 2.** Stages of bibliometric analysis.

where h-index is equivalent to the maximum number (*i*) of cited publications in a countable set N of journal or author publications with at least *i* number of citations. The h-index, which integrates the number of citations (qualitative scales), and the number of publications (quantitative scales), was used to assess the performance and impact of publications in a qualitative view [70]. This is due to the impact of the h-index in evaluating the quality of research produced by scholars, countries, sources, institutions, etc., as reported by [71]. It is worth noting that all the parameters were not manually calculated as the Scopus database provided them. VOSviewer software 1.6.18 was used to process the data to present the findings. Network and overlay visualization of all keywords occurrences (author and index keywords), co-authorship between countries, authors, and organizations results were obtained using VOSviewer as [72]VOS algorithm described.

Each circle in the network visualization represents a keyword, and the size of the circles or nodes presents the occurrences of keywords, therefore the larger the circle, the more the keyword has been co-selected in the topic of biochar-based compost. The color of the circle indicates the cluster to which a keyword belongs. The distance between two keywords in the visualization suggests topic similarity or relative strength. The shorter distance signifies strong similarities, and the thick line connecting the two nodes, the more occurrences the keywords have [3]. The overlay visualization was used to show the trends in keywords used in the topic. For instance, the gradient color shown on the map, from blue to yellow, reveals the freshness of publications [73] and reveals recently appearing keywords. Before the keyword analysis, the authors standardized the keywords manually because based on [74] different expressions of the same keywords might cause errors in the findings.

## 4. Results

The application of biochar and compost has gained momentum over the years, and therefore, a bibliometric analysis to understand current research trends on the biochar and compost topic is useful to analyze growth trends, most productive countries, journals, research hotspots, and most cited publications.

### 4.1. Annual distribution of publications

To assess the academic influence of authors, the number of publications and citations is measured [75], while the h-index is used to measure the scientific output (publications) and citations (impact) [71]. The results of the number of publications, frequency of citations, and h-index presented in Figure 3 show the data collected on publications on biochar and compost from 2011 to 2021, with a total of 254 publications. Of the 254, 85.43% of the publications were articles (*n* = 217), followed by conference papers. An increase in the number of publications by 97.40% between 2011 and 2021 was observed, with the highest number (*n* = 77, 30.31%) of publications in 2021. In 2021, the highest number were published under the discipline of Agricultural and Biological Sciences (*n* = 40, 15.75%) and environmental Sciences (*n* = 36, 14.20%) and published under the journal of IOP Conference Series Earth and Environmental Science (*n* = 7, 2.76%), and journal of Science and Plant Nutrition (*n* = 6, 2.40%). The results of the growth rate of annual citations showed a zigzag pattern, with a peak reached in 2017, with a corresponding increase in the h-index in 2017. It is worth noting that, after a decline from 2011 to 2014, a sharp increase from 2014 and 2015 in both the number of citations and h-index was observed.

**Figure 3.** Annual publications and citations from 2011 to 2022.

### 4.2. Distribution of countries

The map in Figure 4a was constructed to illustrate biochar and compost research across different countries, using the number of publications. Sixty-two (62) countries contributed to the field of biochar and compost. China was the most impactful and productive country, with a total of 49 of 254 (18.11%) publications, followed by the United States (14.20%), Australia (11.42%), Italy (11.02%), Germany (9.84%), and Pakistan (9.45%). The data on the citations per paper and h-index of the countries with 10 and more publications are presented in Figure 4b. Even though China had the highest number of publications, Germany, Australia, Spain, and Austria had the highest number of more than 50 citations. While China, Australia, Germany, and the USA had the highest h-index of 20, 17, 17, and 15, respectively.

**Figure 4.** Contribution of countries to biochar and compost research. (**a**) Global distribution of publications in biochar and compost research. (**b**) the total number of publications, citations per paper, and h-index of countries with 10 or more publications.

#### 4.2.1. Subject areas

The topic of biochar and compost has been discussed in 20 disciplines, with the top 10 displayed in Figure 5. Most papers were published in *Environmental Science* and *Agricultural and Biological Sciences* (*n* = 130). The third category is the field of *Earth and Planetary Sciences*, with the contribution of 7% (*n* = 27) publications, followed by *Biochemistry, Genetics, and Molecular Biology* (*n* = 19, 5%). All the categories had more or less than 10 publications, with the lowest top three under the subject of *Chemical Engineering*, *Engineering*, and *Multidisciplinary*. An annual publication output showed an exponential trend from the top two subject categories with 130 documents each (*R*^*2*^ = 0.8943 and 0.868). It should be noted that, compared to the Environment Science field, the growth trend in the number of publications under the *Agricultural and Biological Sciences* field showed a continuously increasing trend from 2011 to 2021, respectively, with a sharp increase from 2020 to 2021.

**Figure 5.** Subject area and annual trend of publications on the topic of biochar-based compost from 2011 to 2021.

#### 4.2.2. Priority journals

The results showed that the top four most productive sources with the contribution of 48 publications (18.90%) on biochar and compost are from different publishers (Table 2). Among the top 15 sources, the most influential publisher was Elsevier (i.e. *Chemosphere*, *Science of the Total Environment*, *Journal of Soil Science and Plant Nutrition*, *Journal of Environmental Management*, *Waste Management*, *Agriculture*, *Ecosystems and Environment*, *Applied Soil Ecology*, and *Journal of Hazardous Materials*) as shown by the total contribution of 22.44% (57 publications), respectively. After Elsevier, the second-ranking publisher was mdpi (*Agronomy* and *Sustainability*). Moreover, regarding the number of citations, sources followed the order *science of the Total Environment* (Elsevier, *n* = 1126) > *Journal of Hazardous Materials* (Elsevier, *n* = 539) >, *Agriculture, Ecosystems, and Environment* (Elsevier, *n* = 529) >, *Chemosphere* (Elsevier, *n* = 407), etc. Notably, 80% of the sources were in the quartile in category 1 (Q1), which shows that many papers in biochar compost research were published by high-level journals, while 60% of the sources had a Cite Score above 5.

**Table 2.** Top 15 journals in biochar-compost research.

Journal	P	C	CPP	CS	SNIP	SJR
Science of the Total Environment (*Elsevier*)	17	1126	66.24	10.5	2.015	1.81Q1
Agronomy (*mdpi*)	11	170	15.50	2.6	1.331	0.65Q1
IOP Conference Series Earth and Environmental Science	11	3	0.30	0.5	0.436	0.20
Environmental Science and Pollution Research (*Springer Nature*)	9	246	27.33	5.5	1.114	0.83 Q1
Chemosphere (*Elsevier*)	7	407	58.14	10.1	1.708	1.51 Q1
Communications in Soil Science and Plant Analysis (*Taylor & Francis*)	6	65	11.00	1.7	0.667	0.40 Q2
Journal of Environmental Management (*Elsevier*)	6	195	32.50	9.8	1.888	1.48 Q1
Journal of Soil Science and Plant Nutrition (*Elsevier*)	6	14	2.33	3.6	1.526	0.63 Q1
Waste Management (*Elsevier*)	6	315	52.50	11.5	2.225	1.74 Q1
Agriculture, Ecosystems, and Environment (*Elsevier*)	5	529	106.00	9.0	1.896	1.66 Q1
Applied Soil Ecology (*Elsevier*)	5	337	67.40	6.5	1.369	1.11 Q1
Journal of Hazardous Materials (*Elsevier*)	5	539	108.00	13.4	2.158	1.99 Q1
Scientific Reports (*Springer Nature*)	5	310	62.00	7.1	1.377	1.01 Q1
Acta Horticulturae (*International Society for Horticultural Science*)	4	2	0.50	0.5	0.275	0.16 Q4
Sustainability Switzerland (mdpi)	4	6	1.50	3.9	1.242	0.66 Q1

Note* RO: ranking order; **P**: publication; **C**: citation; **CPP**: citation per paper; **CS**: Cite Score; **SNIP**: source normalized impact per paper; **SJR**: Scimago journal ranking.

### 4.3. Most cited papers on the topic of biochar and compost

Table 2 lists the top 20 most cited publications based on Scopus (C^S^) and Google Scholar (C^GS^) databases, including the year of publication and sources/journals. Based on [76] the analysis of the most cited publications assisted scholars to comprehend internal associations among organizations, countries, and authors. The citation report from both databases was used due to significant reported differences between the citation counts of the two databases [77–79]. The papers were published between 2011 and 2019, with most published papers in 2017. The top four most cited papers based on C and CGS are titled ‘efficiency of green waste compost and biochar soil amendments for reducing lead and copper mobility and uptake to ryegrass’ [80], ‘Biochar application to low fertility soils: A review of current status, and future prospects’ [81], ‘Benefits of biochar, compost and biochar – compost for soil quality, maize yield and greenhouse gas emissions in a tropical agricultural soil’ [82], ‘Effects of biochar compared to organic and inorganic fertilizers on soil quality and plant growth in a greenhouse experiment’ [83]. All these papers were published by different sources (Table 3). Of the top 15 most cited papers, two were published in 2012 by the Journal of Plant Nutrition and Soil Science, with another two published by Agriculture, Ecosystems, and Environment in 2014 and 2015, making these sources the most productive based on the number of citations.

**Table 3.** Top 10 most cited publications.

Author	Year/C^S^	C^GS^	Title of the article	Source
Karami et al.	[80]/400	537	Efficiency of green waste compost and biochar soil amendments for reducing lead and copper mobility and uptake to ryegrass	Journal of Hazardous Materials, 191 (1–3), 41–48
El-Naggar et al.	[81]/354	424	Biochar application to low fertility soils: A review of current status, and future prospects	Geoderma, 337, 536–554
Agegnehu et al.	2016/343	502	Benefits of biochar, compost and biochar – compost for soil quality, maize yield and greenhouse gas emissions in a tropical agricultural soil	Science of the Total Environment, 543, 295–306
Schulz and Glaser	[83]/310	501	Effects of biochar compared to organic and inorganic fertilizers on soil quality and plant growth in a greenhouse experiment	Journal of Plant Nutrition and Soil Science, 175(3), 410–422
Agegnehu et al.	[84]/293	398	The role of biochar and biochar-compost in improving soil quality and crop performance: A review	Applied Soil Ecology, 119, 156–170
Kammann et al.	[85]/263	365	Plant growth improvement mediated by nitrate capture in co-composted biochar	Scientific Reports, 5
Hagemann et al.	[86]/228	275	Organic coating on biochar explains its nutrient retention and stimulation of soil fertility	Nature Communication, 8(1)
Liang et al.	[61]/213	250	Changes in heavy metal mobility and availability from contaminated wetland soil remediated with combined biochar-compost	Chemosphere, 181, 281–288
Liu et al.	[87]/211	364	Short‐term effect of biochar and compost on soil fertility and water status of a Dystric Cambisol in NE Germany under field conditions	Journal of Plant Nutrition and Soil Science, 175 (5), 698–707
Schulz et al.	[88]/196	326	Positive effects of composted biochar on plant growth and soil fertility	Agronomy for Sustainable Development, 33(4), 817–827
Agegnehu et al.	2015/185	275	Biochar and biochar-compost as soil amendments: effects on peanut yield, soil properties and greenhouse gas emissions in tropical North Queensland, Australia	Agriculture, Ecosystems and Environment, 213, 72–85
Schmidt et al.	[89,89]/164	258	Biochar and biochar-compost as soil amendments to a vineyard soil: Influences on plant growth, nutrient uptake, plant health and grape quality	Agriculture, Ecosystems and Environment, 191, 117–123
Lashari et al.	[90,90]/153	223	Effects of amendment of biochar-manure compost in conjunction with pyroligneous solution on soil quality and wheat yield of a salt-stressed cropland from Central China Great Plain	Field Crop Research, 144, 113–118
Xiao et al.	[91]/138	160	Recent developments in biochar utilization as an additive in organic solid waste composting: A review	Bioresource Technology, 246, 203–213
Agegnehu et al.	2016/135	204	Crop yield, plant nutrient uptake and soil physicochemical properties under organic soil amendments and nitrogen fertilization on Nitisols	Soil and Tillage Research, 160, 1–13

Note* RO: ranking order, **Year/C**: citation, **TLS**: total link strength, **CS**: Scopus citation, **CGS**: Google Scholar citation.

### 4.4. Co-keywords analysis

A keyword analysis is a bibliometric method used to present development trends and research hotspots [68; 92] of a single domain by showing subjective words that appear in the literature or keywords frequencies [93]. Based on [94] keyword analysis helps sort out researchers’ interests and research themes. All the keywords with 10 occurrences used in the study topic are presented in Figure 6, and Figures 7a & b. From the network visualization presented in Figure 6, VOS viewer software divided all keywords into four clusters (i.e. red, blue, green, and yellow). Among the four clusters, the keyword ‘soil’ had the third-highest occurrences (94), after the search terms ‘biochar’ and ‘compost’ in the red cluster showed strong connection with the search terms, as shown by the short distance and a thick line connecting the terms (Figure 6). For instance, the keyword ‘soil’ in the red cluster with 94 occurrences is associated with ‘soil amendment,’ ‘soil quality,’ ‘soil nutrient,’ ‘soil fertility,’ ‘soil pollution,’ ‘soil organic matter,’ ‘soil moisture,’ ‘soil property,’ ‘nitrogen,’ ‘phosphorus,’ ‘crop yield,’ ‘maize/*Zea mays*,’ ‘greenhouse gas,’ etc.. In the green cluster, the keyword ‘soil,’ is also associated with ‘soil pollution,’ ‘soil pollutant,’ ‘soil remediation,’ ‘heavy metal,’ ‘contaminated soil,’ ‘adsorption,’ ‘bioremediation,’ etc.. The four clusters show the research hotspots on the topic of biochar-based compost, and these can be divided into four; red cluster: application of biochar and compost as an organic soil amendment for enhanced soil quality, fertility, and crop production; green cluster: co-application of biochar and compost in soils contaminated with heavy metals; blue cluster: the influence of biochar and compost on the microbial community; yellow cluster: the influence of biochar and compost on organic carbon, organic matter, and heavy metal content under certain pH conditions.

**Figure 6.** Network and overlay visualization co-occurrence analysis of all keywords (author and index keywords); of the 2098 keywords, 70 met the threshold of 10 occurrences.

**Figure 7.** Overlay (**a**) and density visualization (**b**) of co-occurrence of all keywords (author and index keywords); of the 2098 index keywords, 70 met the threshold of 10 occurrences.

To help researchers learn the main research trends in the topic, it is important to understand the evolution process of keywords used over the past decades. Hence, the overlay visualization in Figure 7a was constructed using VOSviewer software. The gradient color shown in the visualization, from blue to yellow, reveals recently appearing keywords. The evolution process is shown by the red dotted lines, from blue to yellow circles. For instance, the keywords in blue circles such as ‘carbon,’ ‘carbon dioxide,’ ‘carbon sequestration,’ ‘greenhouse gas,’ ‘soil fertility,’ ‘soil nutrient’ etc., appeared earlier around 2017, while keywords in yellow circles on the left corner of the figure such as ‘soil pollution,’ ‘contamination,’ ‘phytoremediation,’ ‘adsorption,’ ‘arsenic,’ ‘cadmium’ appeared between 2019 and 2020.

### 4.5. Country analysis

As an important form of co-authorship analysis, country co-authorship reflects the communication between countries, including the most influential countries. The co-authorship network and density visualization of countries in Figures 8a, b, and c describe the international scientific collaboration of biochar and compost research publications between 2011 and 2021. From the 67 co-authorship countries, 31 met the threshold of 3 documents and a minimum number of 10 citations. However, some 31 items were not connected; the large set of connected items consisted of 30 countries. VOS viewer divided the countries into 5 clusters, which are shown in different colors in the network visualization (Figure 8b). The most prominent countries of each cluster with a shared output of 65.75% are China, the USA, Australia, Italy, and Germany. Moreover, the publications in the red cluster (Figure 8b) (China, USA, Australia, Czech Republic, Poland, Spain, India, and United Kingdom) had a combined contribution of 60.24%. It should be noted that countries in the same cluster and color indicate their intellectual associations with each other. For example, Indonesia, Malaysia, Iran, and Japan in the purple color with the contribution of 16.14% also indicated their intellectual associations.

**Figure 8.** Density visualization (**a**), network visualization (**b**) and overlay visualization (**c**) country on the topic of biochar compost.

Interestingly, some European countries like Italy, France, Austria, Norway, and Switzerland were in the same cluster (green color), with Ghana, an African country. The density visualization map in Figure 8a was used to understand the most dominant co-authorship countries. The map is available in VOS viewer and used to understand the general structure and present important areas in the map [95], as shown by the red and yellow colors. The collaboration between the most dominant countries in different clusters was made clear. For instance, the red to yellow color shows the strong collaboration between China, the USA, Pakistan, and the Czech Republic. Even though China had the highest record of publications, Germany, followed by Australia had the highest number of citations (Table 4). On the other hand, New Zealand, and Switzerland had the highest average citation per publication, and have an average publication year between 2016 and 2017, respectively.

**Table 4.** Country co-authorship on biochar and compost research.

Country	C	P	AC/P	TLS	APY
Germany	2219	25	88.80	38	2016.92
Australia	2095	29	72.24	40	2017.59
China	2056	49	41.96	41	2018.61
USA	1549	36	43.03	41	2018.61
Italy	1118	28	39.93	26	2018.75
Switzerland	905	9	100.56	21	2016.78
Pakistan	788	24	32.83	39	2019.83
Austria	748	14	53.43	22	2017.43
Spain	742	12	61.83	15	2017.75
United Kingdom	594	7	84.86	9	2016.43
South Korea	520	6	86.67	14	2018.67
India	462	7	66.00	9	2019.00
New Zealand	433	4	108.30	11	2017.75
Egypt	413	10	41.30	10	2020.20
France	221	14	15.79	16	2019.36

Note* RO: ranking order, **C**: citation; **P**: publication; **AC/P**: average citation per publication; **TLS**: total link strength; **APY**: average publication.

## 5. Discussion

Out of 16 subject categories, the mainstream research on the research topic was in Environmental science and Agricultural and Biological Sciences, and based on the analysis of all keywords (author and index keywords), the mainstream research was centered on biocharcompost, and co-composted biochar as a soil amendment to improve ‘soil fertility,’ ‘soil quality,’ and for remediation of soil contaminated with inorganic contaminants, with more recent research hotspot on ‘soil pollutants’ (e.g. lead and arsenic) (Figure 7A). Investigations on the effect of biochar and compost mixture on soil quality have shown that they can be applied under different soil conditions. For example [96], investigated the effect of co-application of biochar and compost into a saline soil as an amendment on the growth of roselle (*Hibiscus sabdariffa L*.), and soil quality and reported a significant increase in soil microbial biomass carbon and N, increased N (16%), P (38%), and K (15%) phosphatase, and dehydrogenase activity compared to the control treatment with soil alone. Also, the combined application of biochar and compost in their study, increased the roselle shoot uptake of P, N, and K, by 31, 20, and 25%, including plant height, dry weight, fresh weight, chlorophyll content, etc., compared to the control treatment, and therefore, concluded that biochar and compost mixture increased soil and roselle quality. Using co-composted biochar under saline soil conditions to investigate its effect on soil quality and plant growth [43], reported positive effects on eggplant (*Solanum melongena L*.) growth, increased soil organic matter, N, P, K, water-holding capacity, field capacity, useful pores, available water, and several bacteria in the soil, including reduced bulk density, pH, and electrical conductivity (EC) at different co-composted biochar application rates (0, 5, and 10 t ha^−1^), and irrigation regimes (100, 80, and 60% of evapotranspiration rate).

The most studied crop was maize (*Zea mays*), as a keyword it appeared more than 10 times in several studies on the topic [97; 98]; Adejumo et al., 20221 [36]. In these studies, maize was grown under different soil types to enhance its growth, yield, soil health, soil quality, and fertility. In one study conducted in Ghana by [99] maize is a staple cereal crop that is widely grown in Sub-Saharan Africa [100], and is limited by soil contamination, drought, poor soil fertility, salinity, and excessive heat was grown on industrial soils contaminated with Pb (53, 752 mg kg^−1^), under different light intensities and biochar-compost mixtures (0, 2.5,5, 7.5 t ha^−1^). The authors reported increased yield and vegetative growth of maize under reduced light intensity. These studies show that biochar and compost mixture is a promising soil organic amendment that can be exploited to produce maize under unfavorable and degraded soils.

Another keyword that was linked to ‘soil,’ in the network visualization shown in Figure 6 was ‘greenhouse gas,’ this keyword was used earlier in the research of biochar and compost, based on the overlay visualization (Figure 7a). From the studies retrieved from the Scopus database [82,84,101,102], focused on the effect of biochar and compost applied on acidic Ferralsol and Nitisol on crop yield, soil quality, and greenhouse gas emissions (i.e. CO_2_ and N_2_O) and concluded that biochar-based compost application to acid soils can enhance soil nutrient status, soil organic carbon, soil water content, crop yield, and can help reduce GHG emissions. Also, the effect of biochar and compost on peanut yield and greenhouse gas (GHG) was investigated in Australia on a Ferralsol [103]. It was reported that the mixture could enhance soil health, improve peanut productivity, and reduce GHG.

Out of 62 countries, involved in biochar-compost research, and 67 co-authorship countries based on VOSviewer analysis, China was the most influential country on the topic as shown in Figures 4a, b, and Figure 8a, b, and c. The contribution by China was also noticed in the record of citations, with as 20% of the publications being among the most cited papers on biochar compost (Table 3). The results of co-authorship showed geographical barriers, as China had collaborations with the USA, Australia, Czech Republic, Poland, Spain, India, and United Kingdom, with a collective contribution of 60.24%. An increase in the number of publications from 2011 to 2021, with an anticipated increase in the number in 2022, shows that the research on biochar compost is still growing and is being explored by researchers from different fields of study, and countries or regions. The increasing attention can be explained by the effect of steady and continuous application of inorganic fertilizers on plant accumulation of heavy metals, decreasing grain quality and nutrition of crops [104; 105], including water, air, and soil pollution through the accumulation of toxic chemicals in water bodies, and physical soil degradation [106]. Contrary to the long-term application of inorganic fertilizers, biochar-based compost has proven to be an effective organic fertilizer for soil heavy metal immobilization. For example [61], investigated the effect of biochar and compost applied at different ratios on the speciation distribution and availability of Cu Cd, and Zn in wetland soil. The authors reported decreased Zn and Cd availability in all treatment combinations and associated their findings with increased pH of wetland soil, however, increased Cu contented because of high initial Cu content present in the compost (i.e. 2.25 mg kg ^−1^) and increased water extract organic carbon.

## 6. Conclusion

The properties of the Bibliometric analysis were employed in the present study to investigate current and research trends on the topic of biochar-based compost and co-composted biochar. From the analysis of the 254 publications retrieved from the Scopus database, the number of publications significantly increased between 2011 and 2021, with an anticipated increase in 2022. With China’s collaboration with the USA and other European countries being the top productive country, more collaborations, and funding with African countries, will also help increase the knowledge and benefits of using biochar-based compost and co-composted biochar in most degraded African soils.

## 7. Limitations and suggestions

Like other bibliometric studies, the current bibliometric review has associated limitations. One database (i.e. Scopus) was used to retrieve data, in which a limited number of keywords were used. Therefore, future studies on the topic are recommended to explore different databases, and keywords to avoid missing important publications that are indexed in other databases.
